# Revisiting the regional sustainable development from the perspective of multi-system factor flows–Evidence in the Yangtze River Delta of China

**DOI:** 10.1016/j.heliyon.2023.e18893

**Published:** 2023-08-03

**Authors:** Cheng Shen, Xinyi Zhang, Xiang Li

**Affiliations:** a Shanghai Tongji Urban Planning and Design Institute, Shanghai, 200433, China; b School of Design and Architecture, Zhejiang University of Technology, Hangzhou, 310014, China

**Keywords:** Yangtze River Delta, Multi-system factors, interaction network, Interrelationships, Regional sustainable development

## Abstract

With the advancement of globalization and the interactions between cities globally, the region becomes a basic unit to break through the bottleneck of development and it is becoming a complex system that is inseparable from diverse factor flows. These flows reflect the interaction and can facilitate complementary advantages between cities but will also result in the unreasonable allocation of resources and unbalanced development. To achieve sustainable integration among cities within a region, different factor flows require high-frequency exchange while forming a coordinated effect. This research takes the Yangtze River Delta of China as the research scope, using geospatial analysis, social network analysis, and quantitative statistical analysis methods, selecting representative factor flows such as personnel, information, technology, and capital from 2010 to 2019 to observe the development and integration process within this region. It mainly discusses the development trend, spatial structure and differences of factor flows, the evolution of regional interaction networks, and the interrelationships of different factors to summarize the overall development process comprehensively and find some points that are not conducive to regional sustainable development from the perspective of interaction degree and coordinated effect by some indicators. The research explores a representative and densely populated region in China to provide certain references for regions worldwide through some policy implications.

## 1 Introduction

Since the economic reform and opening-up in China, important progress has been made in developing the factor markets [1]. As the main body promoting urbanization in the age of globalization, the region becomes the basic unit for the allocation of those multi-system factors [2], represented by personnel, technology, information, capital, and so on [3]. These factors form flows among cities within the region which reflect the interaction of multiple resources in the regional development process [4]. Those intercity exchange of factors can facilitate complementary advantages between cities, but it can also result in the unreasonable allocation of resources and uneven development [5]. Thus, these flows can to some extent characterize the comprehensive development status of this region and the interactions across natural and administrative boundaries prompted the evolution trend of regional structure from the center mode to the point-axis mode and then to the network mode, from “space of place” to “space of flow” [6]. In addition, analyzing factors during the interaction process is crucial for promoting regional sustainable development and can help policymakers and urban planners achieve coordinated regional development [7]. To achieve sustainable integration among cities within the region, different factor flows require high-frequency exchange while forming a coordinated effect [5]. Thus, in the period of economic globalization and regional integration, the studies on regions based on the “space of flow” and studies on regional sustainable development should pay more attention to multi-system factor flows with time dimensions and analyze their evolution process, coordinated effect, and interrelationships to find some problems that are not conducive to regional sustainable development.

This research takes the Yangtze River Delta in China as the research scope, selecting representative factors, using multiple methods to analyze the development process of multi-system factor flows comprehensively and find some points that are not conducive to regional sustainable development from the perspective of development balance, interaction degree and coordinated effect by some indicators. The research can provide certain references for the sustainable development of regions worldwide through some policy implications and to some extent supplements the studies on regional sustainable development.

## 2 Literature review

The theory of “Space of flow” was first proposed by Manuel Castells in his book The Rise of the Network Society. He believes that society is constructed around capital, information, technology, and organizational interaction [8]. On this basis, scholars first focused on traditional measured flow data on infrastructure, business investment, and transnational migration. For instance, Goei uses commuter data to analyze the polycentric structure of the greater south-east of the United Kingdom [9]; Limtanakool uses traffic survey data from the Netherlands to measure the evolution of regional network structure [10]; Grady uses the location of American bank checks to reflect people's mobility [11]; Oort analyzes city interactions by using enterprise data from the Ranstad region of the Netherlands [12]. Meanwhile, there are also some studies on regional transportation networks based on high-speed railway data [13], invention patent data [14], and enterprise data [15] in the Yangtze River Delta. This kind of studies mainly measures the urban network structure and urban grade division and especially pay attention to the content of the transportation system [16,17]. Recently many scholars have also analyzed the characteristics of the interaction network structure more deeply based on population flows, information flows, and financial flows [[18], [19], [20]]. However, these studies mostly focus on a single or one kind of factor flow but pay less attention to multi-system or multiple factors and their coordinated effect or interrelationships.

In recent years, with the development of information technology, mobile phone data, internet data, and other big data can enrich the content of this field and make it possible to extend research into cyberspace. For instance, Ratti captures a month's worth of mobile phone data for the UK (excluding Northern Ireland) to measure city interactions [21]; Sobolevsky uses telephone data from seven countries to map the region's hinterlands [22]; Blondel divided Belgium into 17 regions based on six-month telephone records of 2.6 million people [23]. Doran analyzed 2.079 billion mobile phone calls recorded at 1,666 base stations across Senegal over 12 months as a stream of information [24]. In recent years there has been an emerging exploration of using new data, such as GPS data [25], Bluetooth data [26], and internet data from various social platforms [27]. The factor flows generated by new technologies are bound to be different in development characteristics from traditional factors and are free from the constraints of material conditions. At the same time, the coordinated effect between them is also worthy of attention.

Research on regional sustainable development mainly explores areas such as land resources and environmental protection [28,29], industrial and economic development [30,31], government institutional mechanisms [32], and transportation and infrastructure [33,34]. Recently, some scholars have paid attention to the spatial distribution differences of cities’ sustainable development degree in the region and the driving effects of regional sustainable development [35]. Some scholars have also used various flows to explore the coordinated development of regions and their optimal agglomeration pattern [36]. In general, there are still few studies exploring regional sustainable development from the perspective of coordinated effects and interrelationships among multi-system factor flows during an evolution period.

## 3 Materials and methods

### 3.1 Research goal

Against the backdrop of the literature review, the goal of this study is to select a representative region in China, focusing on multi-system factor flows such as personnel, technology, information, and capital and based on the time dimension of 2010–2019, to systematically analyze the evolution characteristics and development process as well as their interrelationships with the comprehensive method and find some problems that are not conducive to regional sustainable development from the perspective of interaction degree and coordinated effect by some indicators and then provide some policy implications on regional sustainable development.

### 3.2 Research scope

The range of the Yangtze River Delta has undergone certain changes, in 2020, China's “Yangtze River Delta Regional Integration Development Plan” officially defined its boundary as Shanghai, Zhejiang Province, Jiangsu Province, and Anhui Province [37]. This research selects all 41 cities in the Yangtze River Delta of China as the research scope which is shown in Table 1. This region represents the strongest and most active economic development as well as a demonstration area for regional integrated development with the most concentrated factors in China [38]. Since 2010, various types of modern infrastructure in this region have been continuously improved and the factor flows among cities in this region have been strengthened steadily.

**Table 1:** Research scope: all 41 cities in the Yangtze River Delta of China.

Province/Province-level municipality	City
Shanghai	Shanghai
Zhejiang Province	Hangzhou, Ningbo, Wenzhou, Shaoxing, Huzhou, Jiaxing, Jinhua, Quzhou, Taizhou, Lishui, Zhoushan
Jiangsu Province	Nanjing, Wuxi, Xuzhou, Changzhou, Suzhou, Nantong, Lianyungang, Huaian, Yancheng, Yangzhou, Zhenjiang, Taizhou, Suqian
Anhui Province	Hefei, Wuhu, Bengbu, Huainan, Maanshan, Huaibei, Tongling, Anqing, Huangshan, Fuyang, Suzhou, Chuzhou, Liuan, Yicheng, Chizhou, Haozhou

### 3.3 Research framework

This research selects personnel, information, technology, and capital factors in the Yangtze River Delta region as the research object. These representative factors in the factor market can largely reflect the comprehensive development status of the region.

The study first analyzes the development process, distribution characteristics, and interaction networks of various factors with geospatial analysis and social network analysis methods among the core city Shanghai, provincial core cities (provincial capitals: Nanjing, Hangzhou, Hefei), megacities (Suzhou, Wenzhou, Ningbo, Xuzhou with a population of more than ten million), large cities (Nantong, Suzhou, etc. With a population of five to ten million) and other cities [39], and compare their differences between regions and provinces. Then combined with the indicators such as network density, centralization degree, and cohesive subgroup degree, the unbalanced characteristic and development problems of networks for factors can be concluded as well. In the second part, QAP (quadratic assignment procedure) method is used to explore the interrelationships and mutual influences of different factors and examine their coordinate effect. By the analysis above, some understandings of regional development from the perspective of multi-system factor flows can be concluded and some policy implications of regional sustainable development based on factor allocation can be proposed.

### 3.4 Data and methods

The source of the data for the personnel factor is the frequency of passenger railway trains between cities in the Yangtze River Delta from 2010 to 2019. The data from 2010 to 2016 was obtained from the “National Railway Passenger Train Schedule” published by China Railway Press and data from 2017 to 2019 are provided by Shanghai Railway Bureau. Each piece of data is the number of trains between two cities per day. After statistics and classification, a 41*41 matrix with a single city as a node is constructed, and then all of them are imported into Ucinet software for network processing to obtain the personnel network dataset.

The data used to analyze the information factor is the annual average of the search index among cities in the Yangtze River Delta from 2010 to 2019. The data is obtained through the Baidu Index interface with the name of each city as a keyword and classified by regions [40]. Each piece of data is the number of mutual searches between two cities per day. Use the same processing method to obtain the information network dataset.

The data used to analyze the technology factor is the annual number of patent cooperation between cities in the Yangtze River Delta from 2010 to 2019. Through the China Patent Information Center of the State Intellectual Property Office, the original data such as the filing date, the applicant, and the applicant's address can be obtained [41]. After processing, each piece of data represents a patent cooperation between two cities.

The data used to analyze the capital factor is the relationship between listed companies’ headquarters and their branches in the Yangtze River Delta. Based on the registered enterprise database of 2010–2019 on the State Administration for Industry and Commerce of China, the headquarters location and numbers of their branches in different cities can be obtained [42]. Each piece of data is a record of where a branch of an enterprise is located. A sample for the dataset of capital factor is shown in Table 2.

**Table 2:** The dataset for capital factors among cities in the Yangtze River Delta (2018).

	Shanghai	Hangzhou	Nanjing	Hefei	…	Wenzhou	Quzhou
Shanghai	–	205	110	67	…	46	15
Hangzhou	205	–	35	18	…	23	19
Nanjing	110	25	–	30	…	1	0
Hefei	67	18	30	–	…	3	1
…	…	…	…	…	…	…	…
Wenzhou	46	23	1	3	…	–	0
Quzhou	15	19	0	1	…	0	–

In the first part of the analysis, combined with the geospatial analysis method, the social network analysis method is used to quantitatively study the interaction network characteristics and dynamic evolution process of factors in the region. Social network analysis is a quantitative method based on mathematical graph theory which describes the structural characteristics of a network comprehensively and objectively through a series of indicators of relational data. This study uses Netdraw software to visualize the network map into the regional spatial layout and summarize the evolution rule of network structure from multiple perspectives through the indicators such as network density, centralization degree, and cohesive subgroup degree.

(1) The network density reflects the overall correlation between nodes in the network and the degree of network development. The higher the value, the stronger the communication and interactive ability of the network. The calculation method is shown in Equation (1) as follows:

(1) $$D=\frac{\sum_{i=1}^{n}*\sum_{j=1}^{n}T_{ij}}{N},i\neq 1$$

Where D is the density of the urban network, $T_{ij}$ is the sum of flows between cities, and N is the number of urban nodes in interaction networks.

(2) Centrality is an index used to judge the influence of each node in the network and the degree of centralization of the overall network. In this study, the centralization degree is selected for evaluation. The lower the value, the more uniform the distribution of nodes in the network; otherwise, the overall structure is not balanced. The calculation method is shown in Equation (2) as follows:

(2) $$C_{i}=\sum_{i=1}^{n}T_{ij}$$

Where $C_{i}$ represents the centralization degree of the city i. And then the calculation method for centralization degree is shown in Equation (3) as follows:

(3) $$C=\frac{\sum_{i=1}^{k}\left(C_{\max}-C_{i}\right)}{\max\sum_{i=1}^{k}\left(C_{\max}-C_{i}\right)},i\neq 1$$

The value ranges from 0 to 1. The lower the value is, the more balanced the network is; otherwise, there is an obvious central node in the network and thus the structure is not balanced.

(3) The cohesive subgroup degree is a technical index to measure the internal structure of the whole network, which is calculated in Equation (4) as follows:

(4) Index(E−I)=(El−IL)/(EL+IL)

where EL represents the number of relationships between subgroups, IL represents the number of relationships within subgroups. Its value ranges from −1 to 1. The closer the value is to 1, the more branch structures with dense interactions exist in the region and there are more metropolitan areas.

In the second part, combined with the results of the first part, the coordinate effect among the different factors is studied quantitatively with QAP (quadratic assignment procedure) to find out their interrelationships. QAP is a research method to test the relationship between matrices based on data replacement. By replacing each value in the two matrices, the correlation coefficient between the matrices is compared to the test, and the coefficient is examined by a non-parametric test. In this study, each factor is used as the dependent variable for regression analysis to test its correlation with different factors. Firstly, the conventional regression analysis is carried out for the long vector corresponding to the independent variable matrix and the dependent variable matrix. Then, the rows and columns of the dependent variable matrix are randomly replaced several times, and the regression analysis is carried out again to get the calculated coefficient and the value of the decision coefficient $R^{2}$.

## 4 Discussion

### 4.1 The evolution process and network structure of multi-system factor flows

Transportation infrastructure is an important spatial channel and direct carrier for the personnel factor, and regional railway transportation has become one of the main ways for people to travel between cities in the Yangtze River Delta, especially after 2010.

As shown in Fig. 1, Fig. 2, the total flows of personnel factors have increased significantly with a long-term sustained and stable trend. The number of flows has rapidly increased from more than 15,000 in 2010 to more than 45,000 by the end of 2019, an increase of 200% in 10 years with the average annual growth rate remaining at 13%. From the perspective proportion accounts for total flows, large cities account for a dominant proportion and show an upward trend. The proportion of large cities with a population of more than five million (about 45% of all cities) has reached 70% and is relatively stable over time. The top eight megacities accounted for nearly 50%. Shanghai, Nanjing, Hangzhou, and Hefei account for nearly 30% and showed an increasing trend from 25.8% to 30.5%. Large cities are still the main participants of personnel factors.

**Fig. 1:** Total flows of personnel factor.

**Fig. 2:** The proportion accounts for total flows.

As shown in Fig. 3, the spatial coverage of the personnel factors has gradually expanded, and the regional structure has an obvious trend of networking. From 2010 to 2019, the strength and density of personnel flows increased significantly, especially the direct interactions between core cities. It can also be seen that flows in cities located on the edge of the region are relatively weak, especially in northern Jiangsu and northern Anhui province, which only rely on the Beijing-Shanghai high-speed railway to carry personnel flows. The flows between large cities have been significantly enhanced, and the network structure has gradually developed from monocentric to polycentric. The flows between Shanghai and the provincial capitals have been significantly enhanced and gradually develop into a network among Shanghai, Nanjing, Hangzhou, and Hefei. At the same time, relying on the transportation trunk lines, the urban nodes (such as Xuzhou, Bengbu, and Wenzhou) located in the transportation hubs also form high-intensity personnel interactions with the core cities.

**Fig. 3:** The evolution of the interaction network of personnel factor in the Yangtze River Delta from 2010 to 2019.

Overall, there are obvious differences in different areas and the development of personnel factor in the region is not balanced. For instance, the flows present differentiated characteristics within each province. The interactions in Jiangsu Province are mainly concentrated along the Shanghai-Nanjing Railway. However, the interactions between the northern cities in this province are weak. The flows in Zhejiang Province show relatively balanced characteristics and the flows in Anhui Province are mainly distributed around the provincial capital.

As for the information factor, the Yangtze River Delta is the first region in China to start the construction of mobile Internet and by 2017, many cities in the region had basically achieved full coverage of 4G networks and then took the lead in starting the application of 5G technology.

As shown in Fig. 4, Fig. 5, the total flows of information factor have doubled, with an average annual growth rate of 9.8% and with the largest increase between 2012 and 2015. The number of mutual searches between cities has increased from 24,000 to more than 50,000, reaching a peak of 52,000 in 2016. The proportions of information flows in all kinds of cities are relatively balanced. Core cities which took the lead in developing the mobile Internet, occupy a dominant position accounting for about 20%. The proportion of large cities is slightly larger than that of small and medium-sized cities, and this proportional relationship has been stable over time which shows that all kinds of cities are in a relatively equal position in the network of information factor.

**Fig. 4:** Total flows of information factor.

**Fig. 5:** The proportion accounts for total flows.

As shown in Fig. 6, the information flows present a relatively stable network structure. From 2010 to 2019, the flows develop from only among some cities in Shanghai, southern Jiangsu, and northern Zhejiang into a network covering most cities, forming a stable network structure that is also composed of several clusters with similar structures. There are stable interactions among small cities, as well as large cities, but the interactions between these two kinds of cities are weak. The overall structure develops from an initial point-axis mode to an obvious polycentric mode.

**Fig. 6:** The evolution of the interaction network of information factor in the Yangtze River Delta from 2010 to 2019.

The structure is relatively balanced. The intensity of flows around Shanghai and in Zhejiang Province is relatively high. The interactions between cities along the Nanjing-Shanghai line in Jiangsu Province are relatively active, gradually radiating to the northern areas. Overall, the structure tends to be more balanced, and the differences and unbalances are mainly reflected between different kinds of cities.

For the technology factor, as shown in Fig. 7, Fig. 8, the total flows have increased periodically. Since 2010, the flows among cities have rapidly increased from 4000 to nearly 24,000, with an average annual growth rate of 23.45%, which is concentrated among large cities and not evenly distributed. Large cities, especially core ones, account for a higher proportion. In 2010, large cities with a population over five million (about 45% of all cities) take up nearly 90% of all flows and the top eight megacities accounted for more than 66%. From 2010 to 2019, the proportion of flows between large cities has declined while small cities are accelerating their integration into regional innovation cooperation networks.

**Fig. 7:** Total flows of technology factor.

**Fig. 8:** The proportion accounts for total flows.

As shown in Fig. 9, the networking degree is weak and the network is still in the initial stage. High-intensity flows concentrate among core cities and only a few cities in each province have formed stable interactions, mostly with core cities, and the interactions between them are weak. The structure is in the transition period from the point-axis mode to the networking mode. The interactions between Shanghai and the provincial capitals are active and present a monocentric structure which means that technological exchanges between Shanghai and surrounding cities are dominant.

**Fig. 9:** The evolution of the interaction network of technology factor in the Yangtze River Delta from 2010 to 2019.

Overall, the structure is not balanced as well. The flows in Jiangsu and Zhejiang are relatively active. The southern part of Jiangsu has high-intensity flows, and the central and northern parts are also growing rapidly while the flows in Anhui Province are mainly concentrated in the surrounding areas of the provincial capital.

For the capital factor, as shown in Fig. 10, Fig. 11, since 2010, the flows have maintained stable growth and the number among cities has steadily increased from 3500 to more than 8500 with an annual growth rate of about 12%. Capital flows between large cities continue to increase, but interactions between core cities have relatively weakened. Large cities have always accounted for a large proportion and show an upward trend: the proportion accounted for by cities with a population of more than five million (about 45% of all cities) has increased from 80% to 83%. However, the proportion of core cities such as Shanghai, Nanjing, Hangzhou, and Hefei has declined, from 45% to 43%. It shows that the capital factors are gradually spilling over from the core cities.

**Fig. 10:** Total flows of capital factor.

**Fig. 11:** The proportion accounts for total flows.

As shown in Fig. 12, since 2010, the structure is becoming networked, and the coverage has continued expanding. It initially gathered around the core cities and gradually spread out to the north and south wings, forming a networking structure. With the continuous increase of the total capital flows, stable economic interactions have been formed among the core cities, the economic network gradually extends to the hinterland of each province, and many small and medium-sized cities form direct interactions with core cities. Besides, the intensity of the interaction between large cities has increased, showing a differentiated polycentric characteristic. At first, capital flows were only formed between Shanghai and the provincial capital cities. As time develops, core cities gradually established an interconnected network.

**Fig. 12:** The evolution of the interaction network of capital factor in the Yangtze River Delta from 2010 to 2019.

Overall, the structure is relatively balanced. Small and medium-sized cities in the three provinces have gradually formed stable interaction with core cities, and the flows in cities closer to Shanghai and the provincial capital is becoming more active. At the same time, the internal structure of each province has certain differences: the flows are balanced in Jiangsu and Zhejiang, while unbalanced in Anhui Province.

### 4.2 The characteristics of interaction networks of multi-system factors

As shown in Fig. 13, interaction networks of all factors have some similarities according to three indicators, the network density continues to increase showing that the networks’ structures are all becoming tighter. In terms of network centrality, although there are some slight differences, the centralization degrees gradually approach, the network extension and complement structure have certain similarities, the hub nodes are similar, and the gaps between urban nodes of different levels are gradually narrowed. In terms of internal structure, the cohesive subgroup degrees also have a similar trend showing that the internal subgroup gradually breaks through the administrative boundary, forming polycentric networking structures.

**Fig. 13:** Network density, centralization degree, and cohesive subgroup degree for different networks of personnel, information, technology and capital factors.

In terms of the trend of changes, the trends of information factor, technology factor, and capital factor are similar, but there are great differences in personnel factor. For network density, information, technology, and capital all show a trend of rapid increase, while personnel factors have weak growth, indicating that the transportation system has already become mature. In the aspect of network centrality, only the personnel factor shows an upward trend, while the rest show a fluctuation decline, indicating that the construction of the transportation network enhanced the status of urban nodes to a greater extent which exacerbates unbalanced. In terms of internal subgroups, the personnel network changed from −0.2 to 0.3, while other factors fluctuate between 0.5 and 0.7, showing that the flows of personnel factor are more dependent on railway transportation and have a weaker influence on surrounding cities. The network of personnel factor is relatively closer to a point-axis mode, while the networks of the other three factors are more balanced.

At the same time, different factors have formed some unique characteristics. Since 2010, the indicators of the information factor have changed the most, the technology factor is also obvious, but the personnel and capital factors have changed modestly. The most significant change in information networks occurred from 2012 to 2015, with the popularization of 4G. The technology factor, however, had a weak foundation while the personnel and capital factors have formed a stable development trend.

As shown in Fig. 14, through the analysis of the change frequency of the network indicators for each factor, it is found that the change ranges of information and technology factors are large, while the ranges of personnel and capital factors are relatively stable. Considering the process of infrastructure construction in the Yangtze River Delta, in terms of response speed, personnel, and information factors are directly affected by the infrastructure and have a fast response speed while the technology factors are slightly slower, and capital factors usually form the corresponding adjustment after other factors have changed. In addition, the changes of each factor show a certain periodicity, usually 3–4 years as a cycle, and finally reach a stable development stage.

**Fig. 14:** The changes in the frequency of the indicators for different factors.

### 4.3 Analysis of the interrelationships among different factors

Taking each network matrix as the dependent variable to calculate the relationship with other networks, the results show that the adjusted $R^{2}$ is mostly between 0.3 and 0.4, indicating that the model is suitable to explain the correlation among factors. It is worth noting that in the model with the personnel network as the dependent variable, the adjusted $R^{2}$ value is generally low, indicating that its correlation with other networks is relatively weak.

As shown in Fig. 15, in the model with the capital factor as the dependent variable, the information factor has a strong influence, the influence of the technology factor remains in a relatively stable range, while the influence of the personnel factor is weak, and its influence will be increased only when there is an important transportation trunk completed. In the model with the technology factor as the dependent variable, the information factor has a strong influence, while the capital factor has a stable influence on it, which fluctuates in a small range but shows an overall upward trend. However, the influence of the personnel factor is weak, and its influence will rise only when the regional transportation structure has a huge adjustment. In the model with the personnel factor as a dependent variable, other factors have little influence on it and the influence of technology factors fluctuates greatly. In the model with the information factor as the dependent variable, the influence of technology and capital factors is almost the same, while the influence of the personnel factor is always at a low level. It indicates that the economic and technological innovation of a city in the information age greatly impacts its attraction to the Internet.

**Fig. 15:** Regression analysis with personnel, capital, information and technology factors as dependent variables respectively based on the QAP method.

## 5 Conclusion

In terms of the overall developing process, the flows of personnel, information, technology, and capital factors show a continuous growth trend in the Yangtze River Delta from 2010 to 2019. While the total amount has achieved substantial growth, it has also maintained a fast growth rate, demonstrating a future of high-frequency exchange of factor flows within this region. On the whole, larger cities (with a population of more than five million) account for a larger proportion of flows with faster growth, occupying a dominant position, while other cities are relatively weakly interacting with each other. Meanwhile, the main direction of the flows in these small and medium-sized cities is also Shanghai and provincial capital cities, indicating that the regional structure still has a strong centrality and is unbalanced. As time develops, small and medium-sized cities tend to gradually play a more important role since the proportion and growth rate of the flows among them shows a slightly upward trend, especially for the information factor.

Interaction networks of the factors have commonalities in their evolution process, and similarities in terms of spatial structure, network system, and indicators. They all show the significant strengthening of the main structure, gradual extension of the secondary structure, and continuous improvement of the local structure, with the overall network structure becoming tighter and the network density continuing to increase. For network centrality, the central potential degree gradually approaches, the hub urban nodes are similar, and the gap between urban nodes of different levels is gradually narrowed. For internal structure, the internal subgroups gradually break through the administrative boundary, forming a polycentric structure. Besides, the change of each factor shows a certain periodicity, usually 3–4 years.

However, each factor also has certain differences in the network degree of the core structure, the development direction of the secondary structure and local structure, and the changing trends of the indicators. The changing trend of information, technology, and capital factors are similar, but different in personnel factor. For network density, information, technology, and capital all show a trend of rapid increase, while the personnel factor has weak growth. For network centrality, only the personnel factor shows an upward trend, while the others show a fluctuation decline. For internal subgroups, the personnel factor is more dependent on rail transit lines and weakly influences surrounding cities. The network of personnel factor is closer to a point-axis mode, while the networks of the others are more balanced, especially the information factor. The network of information factor has high intensity, relatively low centrality, and more subgroups, gradually breaking through the geographical limitations and forming flows across the administrative boundaries. Other factors, especially personnel factor, are still unbalanced in their network development. The change ranges of information and technology factors are large, while the changes in personnel and capital factors are stable, showing the different sensitivity of factors in the evolution process.

Through correlation analysis among factors, it is found that the information factor strongly influences other factors while technology and capital factors strongly influence other factors but their influence decreases as time develops. The influence of the personnel factor is weak, even occasionally with no significant correlation, indicating that it lacks effective coordination with other factors. The interactions between information, technology, and capital factors all have a certain degree of spontaneity so the development has some similarities. However, the materiality of the transportation network determines the restricting effect of its spatial structure on the free movement of personnel and logistics within the region, so it may not fit perfectly with the natural development trend of the region and has a low matching degree with other factors. On the other hand, the transportation capacity is limited, the personnel flows between some core urban nodes are close to the upper limit while some cities lack high-frequency personnel flows, and the development of transportation infrastructure is unbalanced in the region. The development characteristics of various factor flows are not consistent, maybe different systems have not formed a unified development goal such as future development priorities and structural expansion directions. If there is no policy guidance, it will not be conducive to the in-depth sustainable development of regional integration.

Therefore, in future sustainable regional planning, more attention should be paid to the coordinated effect among factors by improving the layout of relevant infrastructures and policies. Firstly, in response to the information factor with more networked structure and detachment from spatial constraints, other factors, especially personnel factor, should be guided to effectively cooperate with it, and the transportation infrastructure should be balanced and improved. Secondly, we need to guide the development of capital and technology factors in small and medium-sized cities to ensure they can better integrate into the regional network of diver factor flows. Finally, in the later stage of regional development, it is necessary to guide the establishment of factor flows across the administrative boundaries and among different levels of cities, form more secondary structures, make the network more diversified, and better achieve sustainable integration. Future research should consider the potential causes and possible consequences of differences in the development process of diverse factors more carefully and provide exact policy implications for regional sustainable development from the perspective of different factors respectively.

## Author contribution statement

Cheng Shen: Conceived and designed the experiments; Performed the experiments; Contributed reagents, materials, analysis tools or data; Wrote the paper.

Xinyi Zhang: Conceived and designed the experiments; Performed the experiments; Analyzed and interpreted the data; Contributed reagents, materials, analysis tools or data; Wrote the paper.

Xiang Li: Conceived and designed the experiments; Analyzed and interpreted the data.

## Data availability statement

Data will be made available on request.

## Additional information

No additional information is available for this paper.

## Declaration of competing interest

The authors declare that they have no known competing financial interests or personal relationships that could have appeared to influence the work reported in this paper.
